# Research on Compression Sensing Positioning Algorithm of Indoor Complex Environment Visible Light Indoor Based on Hybrid APIT

**DOI:** 10.1155/2022/9832244

**Published:** 2022-04-21

**Authors:** Yi Li

**Affiliations:** School of Information Engineering, Xi'an University, Xi'an, Shaanxi, China

## Abstract

In today's highly urbanized world, indoor space is becoming more extensive and more complex, and under the increasingly urgent needs, indoor positioning has attracted people's attention. With the rapid development of LED lighting technology, indoor positioning technology based on visible light communication has many advantages over traditional indoor positioning technology. Aiming at the influence of environmental factors such as noise and reflected light on the positioning accuracy, the compression perception theory is applied to the localization of visible light. The position of the receiving end in the positioning space is defined as a sparse variable in the discrete space. The power measurement matrix is expressed as the product of the observation matrix, and the sparse matrix and sparse vector in the compression perception theory are expressed. The traditional APIT algorithm is easy to misjudge unknown nodes in the triangle, resulting in low positioning accuracy of the algorithm. In this study, an indoor visible positioning algorithm based on hybrid APIT is proposed, which uses the area relationship of the triangle to determine the initial position of the unknown node, and then uses the tangent circle to further narrow the area where the unknown node may be located, and uses the hybrid centroid localization algorithm to obtain the estimated position of the unknown node.

## 1. Introduction

### 1.1. Background and Significance

In recent years, with the rapid development of the economy and modern science and technology, service based on location information has been widely used in people's daily lives, and location information has become an essential key basic information in everyday life [1]. At present, the global positioning system (GPS) and other satellite positioning systems that have been widely used in outdoor positioning can already achieve high positioning accuracy [2]. Although GPS can achieve high positioning accuracy outdoors, in the indoor environment, which accounts for 80% of a human daily lifetime, due to the blocking of satellite signals by buildings, the GPS positioning accuracy in indoor environments has dropped sharply, which cannot meet people's demand for indoor positioning services. See Figure 1.

Indoor positioning technology plays an important role in public safety, commercial activities, military fields and other fields, in large shopping malls, users can quickly locate the location of the target goods, according to the personal location, and product information for route navigation [3]. In the library, it can help readers quickly and effectively obtain the required book resources, improve the efficiency of book search and service quality. At the scene of a sudden disaster, rescue workers can be helped to rescue trapped people quickly. As a result, indoor positioning has gradually become the focus of attention of researchers in various countries [4].

The shaded area of the tangent circle where the projection point *M* is located.

  Bluetooth positioning: Bluetooth technology is a short-range, low-power wireless transmission technology that measures signal strength for positioning. Bluetooth location technology is easy to integrate into mobile devices such as mobile phones and is ideal for commercial promotion [5]. The disadvantage is that the cost of the positioning system is relatively high, the stability is poor, and the interference information in the indoor environment is considerable [6].
  Radio Frequency Identification (RFID): Determines the use of radio frequency for contactless two-way communication to exchange data bit. RFID propagation distance is short, up to tens of meters. The advantage of RFID technology is that the positioning accuracy is high and the positioning cost is relatively low. The disadvantage is that the positioning distance is relatively short, and it is not easy to mix with other positioning systems [7].

The projection point *M* is located outside the ABC square Δ.

The advantages and disadvantages of common indoor positioning techniques are shown in Table 1.

### 1.2. Research Status of Indoor Positioning Technology Based on Visible Light Communication

Visible light communication (VLC), also known as nm wave communication, is a communication technology that uses the visible light spectrum of 380 to 740 nm as an information carrier. Because LEDs have high efficiency, long life, and fast response characteristics, they are more suitable for wireless communication than other visible light sources.

Compared with traditional radio frequency (RF) wireless communication, VLC has the following advantages:

- VLC has an unlicensed bandwidth of about 400 THz and rich spectrum resources.
- VLC is easy to implement, just install a microcontroller to build a network using existing LED equipment.
- VLC uses visible light as a carrier and will not cause electromagnetic interference to other electronic devices.
- VLC link can easily set up high-speed communication links above 10 Gb/s.

#### 1.2.1. Research Status of Visible Light Communication Technology

LED visible light source, with its ubiquitous, green, and rich spectral resources, has aroused extensive research interest in the field of indoor broadband communication and intelligent lighting [1]]. Since 2000, Japanese researchers have proposed IB communication systems that use LEDs as communication base stations [8]. Later, Japanese researchers found that visible light communication (VLC) has good prospects for development, so they began to invest a lot of human, material, and financial resources for in-depth research. After a series of theoretical research and practical work, researchers at Nakagawa Laboratory in Japan proposed a VLC system based on carrier monitoring of multiple access and conflict detection, which significantly promoted the development of VLC technology [9].

#### 1.2.2. Research Status of Indoor Visible Light Positioning Technology

*(1) Current Status of Foreign Research*. From the current development trend and market share, it is known that the data wireless communication technology based on visible light will have unlimited market prospects in the future. Many scientific research institutes and enterprises in developed countries such as Japan, Europe, and the United States have invested substantial financial, material, and human resources in visible light communications to conduct research in this field. In 2000, Nakagawa Laboratories in Japan first conducted research on visible light communication technology. At the beginning of the research, the staff of the laboratory spent most of their time on the research of communication channel theory, mainly using mathematical analysis and computer simulation methods to explore, and clarified the possibility that white light-emitting diodes can be used as a light source for the development of indoor lighting and communication systems. After two years, the staff of Nakagawa Laboratory achieved many results in the research of channel models. The staff of Nakagawa Laboratory focused on the specific functional part of the visible light communication system. For the research of visible light communication technology, a scientific research plan on visible-light wireless communication technology has been established in Europe and the United States, which is composed of about 20 scientific research groups in Europe, and has carried out a lot of in-depth research in the field of visible light communication. It was founded at the beginning to develop a new communication method that can provide high-speed data transmission. After a long period of research and research, it has achieved relatively fruitful research and development results in this field. In 2009, the famous Professor Brien of the University of Oxford and others successfully developed and designed a large breakthrough in data communication rate based on equalization technology, at which time the communication rate can be obtained by 100 Mbit/s. Good results have been obtained in the study of visible light communication systems. A year later, in 2010, Brien and others at the University of Oxford innovatively proposed multiinput, multiple-output, and quadrature frequency-division multiplexing techniques to double the communication rate by 100 megabits, resulting in a transmission rate of 220 Mbit/s. In addition to the abovementioned foreign research team, UC-Light, which relies on the University of California and the National Laboratory of the United States, is also one of the essential institutions for visible light communication research, and researchers at the institution have successfully developed an LED lighting system that can achieve high-speed communication and positioning.

*(2) Current Status of Domestic Research*. Compared with foreign countries, domestic research on visible light communication started late. There are still many shortcomings and deficiencies in technology, and there is no mature finished product on the visible light communication system. However, after years of exploration by experts in China, the wireless data communication and positioning system based on visible light has achieved good results in the software method of realizing the principle and the research of the basic physical model of the hardware.

*(3) Overall Situation*. With the advent of the mobile Internet era, emerging technologies are gradually applied to daily life, such as AutoNavi Map, Baidu Map, and other navigation and positioning APPS, and gradually integrated into people's daily lives. GPS can only provide a good positioning effect outdoors, but in complex indoor environments, GPS positioning is more difficult to achieve indoors due to signal attenuation. With this in mind, industry personnel have carried out a lot of research work, and RFID technology, ultrasonic technology, etc., have been applied to indoor positioning systems. Among them, typical cases mainly include RADAR indoor positioning system developed by Microsoft [10].

#### 1.2.3. Application Prospect of Indoor Visible Light Positioning Technology

In today's highly urbanized world, indoor space is becoming more extensive and more complex, and under the increasingly urgent needs, indoor positioning has attracted people's attention. In the past few years, indoor positioning research has mainly stopped at Wi-Fi, RFID, ZigBee, Bluetooth, and other technology fields. In recent years, with the gradual promotion of LEDs in the field of lighting, LEDs are known for their green environmental protection [11].

LED-based visible light positioning technology as a combination of lighting and optical communication, green energy saving, can broaden the spectrum of new wireless communication technology resources, compared with the existing GPS, and radio wave-based positioning technology, with many advantages without electromagnetic interference, high positioning accuracy, especially suitable for a variety of large shopping malls, museums, etc., underground parking, and the large indoor environment with lots of room [12].

For example, at present, the AutoNavi platform is committed to promoting online to offline applications, which can display people, shops, and cars nearby. The method is to achieve outdoor high-precision map positioning, but it cannot achieve high-precision indoor positioning, because according to the above content this can be known only based on visible light wireless data communication indoor positioning technology which can theoretically and effectively achieve indoor accurate two-dimensional and three-dimensional positioning. Therefore, visible light-based wireless data communication indoor positioning technology has incomparable advantages in the future, which can be combined with outdoor positioning technology to achieve seamless positioning of the whole region.

## 2. Visible Light Positioning System Analysis

### 2.1. Diode Basic Principles

A light-emitting diode is a general-purpose lighting device, also known as an “LED,” which is made from a variety of fusion compounds. When the LIGHT-emitting diode is energized, the electrons and holes in its core circuit output visible light through energy radiation. Light-emitting diodes are generally used as indicator lights in electronic devices and can complete digital displays, text displays, or graphic displays. At present, there are three main types of light-emitting diodes: red light, green light, and yellow light. When the internal circuit of the LIGHT-emitting diode has a current flowing through, the “electrons” and “holes” present in it continue to flow through the similar structural surface of the PN junction. This allows them to recombine to produce radiant light spontaneously. Its basic principle is as follows: when the current is directly poured into the light-emitting diode, when the current meets the light-emitting conditions and does not damage the equipment, the light-emitting diode emits normal light, and the main reason is that the light-emitting diode is a semiconductor, and its internal excited electrons are restored from the high-energy level to the low-energy level, and the result of the output are photons as output. When a forward voltage is applied to the PN junction of the LED, it is combined and emitted after the simultaneous injection of a few carriers and most carriers.

### 2.2. Indoor Visible Light Positioning Principle

In the indoor visible light positioning system, the LED lamp is fixed to the ceiling as a signal transmitter to provide illumination during data transmission, led lighting emits a light signal with identification information (ID), the receiver recovers the original signal after processing the collected signal, and then uses the visible light positioning algorithm to calculate the receiver's [13] specific location.

The light intensity distribution of LEDs follows a pattern close to that of Lambert, and typically, we equate all LED illumination lamps with Lambert luminous mode [2®, as shown below:

(1) $$\begin{array}{c} I_{\varphi }=\frac{m+1}{2\pi }{\left(\text{cos }\varphi \right)}^{m}, \end{array}$$

where for the light source radiation pattern, its relationship with the half-power angle emitted by the LED can be expressed as *m*:

(2) $$\begin{array}{c} m=-\frac{\text{ln}2}{\text{ln}\left(\text{cos}\phi_{12}\right)}. \end{array}$$

Modulation characteristics refer to the characteristics of converting electrical signals into optical signals, mainly including three aspects 0]. First, the volt-ampere characteristics of LEDs are similar to those of ordinary diodes, as shown in Figures 2 and 3. When the forward voltage is greater than the on voltage U, then the voltage is proportional to the current.

Define the modulation system of the LED as *m*:

(3) $$\begin{array}{c} m=\frac{1}{2}\frac{\Delta I}{I}. \end{array}$$

Among them, the peak-to-peak current is the AC signal. The larger the modulation system, the easier it is for the receiver to detect the light signal emitted by the LED Δ*I*.

The modulation bandwidth is primarily affected by the device junction capacitance and the lifetime of a small number of carriers in the semiconductor. The 3 dB bandwidth of the LED can be expressed as *f*_*c*_:

(4) $$\begin{array}{c} f_{c}=\frac{3}{2\pi \tau }. \end{array}$$

### 2.3. Channel Characteristics of Visible Light Positioning Systems

In indoor visible light positioning systems, LEDs provide illumination when entering the hall for data transmission. The link mode of its transmission channel can be divided into two categories. The first type is that the optical signal transmission process is not interfered with by the line of sight chain: “The second type is a non-line of sight link that is interfered with during transmission, in which the optical signal emitted by the LED transmitter reaches the receiver after being reflected by obstacles such as ceilings and walls” [14].

According to the Lambert radiation model, the channel gain of the line-of-sight link [3] is

(5) $$\begin{array}{c} H_{d}=\frac{\left(m+1\right)A_{R}}{2\pi d^{2}}{\text{cos}}^{m}\left(\theta \right)\text{cos}\left(\psi \right)T_{s}\left(\psi \right)g\left(\psi \right)\text{rect}\left(\frac{\psi }{FOV}\right). \end{array}$$

In them, the Lambert radiation coefficient, receiving area, field of view, radiation angle of light source, and receiving angle are the straight line distance between the light source and the receiver, for the filter gain at the receiving end, for the gain of the condenser lens at the receiving end, and the rectangular function can be expressed as *mA*_*R*_*FOVθψ*d*T*_*s*_(*ψ*)*g*(*ψ*)

(6) $$\begin{array}{c} \text{rect}\left(x\right)=\left\{\begin{array}{cc} 1, & \text{for}\left|x\right|\leq 1,\\ 0, & \text{for}\left|x\right|>1. \end{array}\right) \end{array}$$

In the model above, the received power at the receiving end can be expressed as follows:

(7) $$\begin{array}{c} P_{r}=H_{d}P_{t}, \end{array}$$

where the average transmit power of the LED transmitter is represented, and the receiving terminal power represents the optical power received by the receiver. In the indoor visible positioning system model, the conversion coefficient of the photodetector is *P*_*t*_*P*_*r*_*η*, which can be expressed as the conversion formula:

(8) $$\begin{array}{c} i_{c}=\eta P_{r}. \end{array}$$

Similarly, the electrical signal power can be expressed as follows:

(9) $$\begin{array}{c} P_{e}=i_{e}^{2}R. \end{array}$$

The relevant positioning system parameters are shown in Table 2.

### 2.4. Reflection Model

Apply the Phong reflection model in the real drawing to indoor visible light positioning to obtain a reflection model that is more in line with the actual positioning environment. Since the optical signal that reaches the receiving end after multiple reflections is far less than the case where direct radiation arrives after a single reflection [1], the reflection model in this article ignores the optical signal that arrives at the receiving end after two or more reflections [15].

The reflection model of the visible light positioning system is shown in Figure 1 [1]. After the LED emits a light signal, it reaches the wall, part of which is absorbed by the reflective surface and the other part is emitted by the wall. We divide the wall into several microreflective surfaces [16], assuming that the micro reflector surface is a receiver with a receiver area, and calculate its received power. Then, each microreflective surface on the wall is an ideal source of Lambert radiation, and the radiation pattern has nothing to do with the angle of incidence of light. In each microreflection surface, the incident light is absorbed by the microreflector surface with the probability of specular reflection, and diffuse reflection occurs with the probability of reflection, and the spatial distribution of the reflected light intensity is *dA*  *dA*1 − *ρρ* · *αρ* · (1 − *α*):

(10) $$\begin{array}{c} H_{ref}=\frac{\rho \cdot \left(1-\alpha \right)}{\pi }\cdot \text{cos}\left(\theta_{2}\right)+\frac{\rho \cdot \alpha \cdot \left(m+1\right)}{2\pi }\cdot {\text{cos}}^{m}\left(\theta_{2}-\psi_{1}\right), \end{array}$$

where the reflection coefficient is the mode parameter of the directionality of the reflected light, and the ratio of specular reflection to total reflection is *ρmα*.

The signal strength received by the receiver after a single reflection through the wall is

(11) $$\begin{array}{c} P_{\text{recerved}}=H_{\text{ref}}\cdot P_{\text{somrce}}, \end{array}$$

where the incident light power of the reflective surface is*P*_*somrce*_.

### 2.5. Noise Model

In a visible light positioning system, the noise component consists of a combination of shot noise and thermal noise *N*:

(12) $$\begin{array}{c} N=\sigma_{th}^{2}+\sigma_{\text{shot}}^{2}. \end{array}$$

The power of thermal noise can be expressed as follows:

(13) $$\begin{array}{c} \sigma_{th}^{2}=\frac{8\pi kT_{c}}{G}\eta A_{R}I_{2}\beta^{2}+\frac{16\pi^{2}kT_{e}\Gamma }{g_{m}}\eta^{2}A_{R}^{2}I_{3}\beta^{3}. \end{array}$$

The power of the shot noise can be expressed as follows:

(14) $$\begin{array}{c} \sigma_{\text{shot}}^{2}=2qRP_{BS}A_{R}\lambda \beta +2qRP_{r}\beta +2qI_{DC}\beta . \end{array}$$

### 2.6. Summary

This study introduces the basic working principle of visible light positioning system analysis and the characteristics of channels and conducts theoretical research on light visible positioning system. It lays the groundwork for the algorithm for indoor visible light positioning methods and common positioning alogrithms.

## 3. Visible Light Positioning Methods and Common Positioning Algorithms

### 3.1. Indoor Positioning Performance Indicators

Different indoor application scenarios will put forward different performance requirements for the system, so the designer needs to design the positioning system according to the actual needs. At present, the performance indicators of the indoor positioning system of visible light communication mainly include the following aspects: positioning accuracy, complexity, system function robustness, functional ductility, and cost [60]: (1) The accuracy of positioning is one of the most important performance indicators based on the visible light wireless data communication positioning technology system, which is to use the average value of the positioning error to estimate the accuracy, the smaller the value, the higher the accuracy. (2) Complexity of hardware equipment requirements and software complexity, which is the critical factor in evaluating manufacturing costs, when the system is complex and redundant, it will cost a lot of costs. (3) Robustness is a key factor in evaluating the performance of indoor positioning systems, and a good system can cope with most bad contingencies. (4) Extensibility is the guarantee of the performance of the positioning system, which can be extended from two-dimensional positioning to three-dimensional positioning, which is the focus of current research in this field. (5) The cost is whether the ratio of the cost and return of the positioning system to the research is reasonable, and the cost of the positioning system is considered from several aspects such as resources, space, time, and cost.

### 3.2. Visible Indoor Positioning Methods

At present, the most widely used visible light indoor positioning methods mainly include the following categories: geometric measurement method, proximity perception method, scenario analysis method, and image sensor imaging method [17].

#### 3.2.1. Geometric Measurements

*(1) RSS Positioning Algorithm*. The RSS positioning algorithm estimates the distance from the receiver to each LED transmitter by measuring the received signal strength at the receiving end, and finally, estimates the position of the receiver by a trilateral measurement algorithm. In the visible light indoor positioning system, each LED emitter emits a light signal with identification information, the receiver determines the source of the optical signal according to the received ID identification information, and finally estimates the distance between the LED transmitter and the receiver according to the received signal strength [18].

*A*(*x*_1_, *y*_1_), and then find the position coordinates of the receiver according to equation (15) and find the position coordinates of the receiver:

(15) $$\begin{array}{c} B\left(x_{2},y_{2}\right)C\left(x_{2},y_{2}\right)\left(x,y,z\right)，\left\{\begin{array}{c} {\left(x-x_{1}\right)}^{2}+{\left(y-y_{1}\right)}^{2}=d_{1}^{2},\\ {\left(x-x_{2}\right)}^{2}+{\left(y-y_{2}\right)}^{2}=d_{2}^{2},\\ {\left(x-x_{3}\right)}^{2}+{\left(y-y_{3}\right)}^{2}=d_{3}^{2}. \end{array}\right) \end{array}$$

*(2) TOA Positioning Algorithm*. A TOA positioning algorithm is required to measure the time it takes for a signal to reach the receiver from the LED transmitter. In a bit-to-position system, when the position information of the three LED transmitters is known, the time it takes for the light signal to reach the receiver from the three LED transmitters is measured separately, and the root (16) is saved, and the time taken for the signal to reach the receiver can be calculated. The distance between LED emitters, in equation (16), is the speed of light. The position coordinates of the receiver are then calculated according to equation (15). *ttt*_1_*,t*_2_*t*_3_*d*_1_*,d*_2_*,d*_3_*c*:

(16) $$\begin{array}{c} d=c*t. \end{array}$$

There are two main problems with the TOA localization method. First, all LED transmitters and receivers must use a fully synchronized clock. Due to the very fast speed of light propagation, if the clock synchronization cannot be guaranteed, the positioning error will be directly generated. Second, the optical signal must contain a timestamp, which reduces the data transfer rate [19].

By measuring the transmission time difference between the signals of different LED transmitters to receivers, determine the distance difference between different LED transmitters and receivers based on the propagation speed of the optical signal. The position coordinates of the receiver are then obtained according to equation (16) *t*_*ct*_*c*.

(17) $$\begin{array}{c} \left\{\begin{array}{c} R_{12}=c\left[\left(t_{1}-t_{r}\right)-\left(t_{2}-t_{r}\right)\right]=c\cdot \left(t_{1}-t_{2}\right),\\ R_{23}=c\left[\left(t_{2}-t_{r}\right)-\left(t_{3}-t_{r}\right)\right]=c\cdot \left(t_{2}-t_{3}\right),\\ R_{13}=c\left[\left(t_{1}-t_{r}\right)-\left(t_{3}-t_{r}\right)\right]=c\cdot \left(t_{1}-t_{3}\right), \end{array}\right) \end{array}$$

where, represents the time when the signal arrives at the receiver from different LED transmitters, the transmission time of the signal, the speed of light, and the LED *t*_1_*,t*_2_*t*_3_*t*_*r*_*cR*_12_*,R*_23_*R*_13_, the distance difference between the transmitter and the receiver. Assume that the position coordinates of the three LED emitters are the sum of the receivers (*x*_1_, *y*_1_), (*x*_2_, *y*_2_)(*x*_3_, *y*_3_).

If the position coordinates are (*x*, *y*), the coordinates of the receiver can be obtained by equation (18):(*x*, *y*)

(18) $$\begin{array}{c} \left\{\begin{array}{c} \sqrt{{\left(x-x_{1}\right)}^{2}+{\left(y-y_{1}\right)}^{2}}-\sqrt{{\left(x-x_{2}\right)}^{2}+{\left(y-y_{2}\right)}^{2}}=R_{12},\\ \sqrt{{\left(x-x_{2}\right)}^{2}+{\left(y-y_{2}\right)}^{2}}-\sqrt{{\left(x-x_{3}\right)}^{2}+{\left(y-y_{3}\right)}^{2}}=R_{23},\\ \sqrt{{\left(x-x_{1}\right)}^{2}+{\left(y-y_{1}\right)}^{2}}-\sqrt{{\left(x-x_{3}\right)}^{2}+{\left(y-y_{3}\right)}^{2}}=R_{13}. \end{array}\right) \end{array}$$

*(3) A0A Positioning Algorithm*. The positioning system based on the AOA positioning algorithm needs to measure the arrival angle of the light signal relative to the LED emitter, and then use the intersection of the direction lines to locate the target. Positioning in 2D space requires two LED emitters, and positioning in 3D space requires at least three LED emitters [20].

In a two-dimensional space, based on the positioning system, the two LED emitters with known position information, now assume that the signal measured by the receiver arrives at an angle of sum, and the coordinates of the receiver are sum, then according to the position coordinates of the LED emitters, A and B can be arranged with a set of equations *A*(*x*_1_, *y*_1_)*B*(*x*_2_, *y*_2_)*φ*_1_*φ*_2_(*x*, *y*):

(19) $$\begin{array}{c} \left\{\begin{array}{c} \text{tan}\left(\varphi_{1}\right)=\frac{y-y_{1}}{x-x_{1}},\\ \text{tan}\left(\varphi_{2}\right)=\frac{y-y_{2}}{x-x_{2}}. \end{array}\right) \end{array}$$

In a two-dimensional space, the optical signal can be processed by using formula (19) to obtain receiver coordinates, owing to the existence of an elevation angle in the actual positioning, resulting in a too large positioning error, so in the actual positioning, the AOA positioning method is rarely used alone, and is usually combined with other positioning algorithms for positioning.

The approximate perception method has the advantages of simplicity, wide coverage, and fast positioning speed. Still, the positioning result of the method is relatively rough. It can only be used as a simple estimation process before positioning. It is necessary to install the LED emitters in accordance with reasonable rules, and the positioning accuracy is highly dependent on the number of LED emitters (21).

#### 3.2.2. Image Sensor Imaging Methods

In the visible light positioning system, the image sensor imaging method is used for positioning, and the lens is mainly placed vertically on the connection line between the LED emitter and the image sensor, so that the three are straight, and the three-dimensional position coordinates of the image sensor are obtained by using their geometric relationship (22).

Compared with the above algorithm, the image sensor imaging method has a higher positioning accuracy, and the higher the resolution of the image sensor, the better the positioning effect. The disadvantage is that the positioning complexity and the price are high.

A description of the two grids near the fence is shown in Figure 4.

### 3.3. RSS-Based Multifaceted Measurement Positioning Algorithm

#### 3.3.1. Introduction to Positioning Algorithms

In an indoor 3D spatial positioning system, LED emitters can be mounted on horizontal planes at different heights and require at least four LED emitters. The receiver can distinguish between light signals from different LED emitting sources by LED-ID identification. The set sum is the position coordinates of the four LED emitters, calculating the distance between each transmitter reaching the receiver based on the received signal strength measured by the receiver and then going through equation (20), lists the systems of equations used to calculate receiver position coordinates. *T*_1_(*x*_1_, *y*_1_), *T*_2_(*x*_2_, *y*_2_), *T*_3_(*x*_3_, *y*_3_)*T*_4_(*x*_4_, *y*_4_)*d*_1_, *d*_2_, *d*_3_*d*_4_*X*=(*x*, *y*, *z*)

(20) $$\begin{array}{c} \left\{\begin{array}{c} {\left(x-x_{1}\right)}^{2}+{\left(y-y_{1}\right)}^{2}+{\left(z-z_{1}\right)}^{2}=d_{1}^{2},\\ {\left(x-x_{2}\right)}^{2}+{\left(y-y_{2}\right)}^{2}+{\left(z-z_{2}\right)}^{2}=d_{2}^{2},\\ {\left(x-x_{3}\right)}^{2}+{\left(y-y_{3}\right)}^{2}+{\left(z-z_{3}\right)}^{2}=d_{3}^{2},\\ {\left(x-x_{4}\right)}^{2}+{\left(y-y_{4}\right)}^{2}+{\left(z-z_{4}\right)}^{2}=d_{4}^{2}. \end{array}\right) \end{array}$$

Conversion to matrix form can be expressed as

(21) $$\begin{array}{c} AX=B, \end{array}$$

where

(22) $$\begin{array}{c} A=\left[\begin{array}{c} x_{1}-x_{2}y_{1}-y_{2}z_{1}-z_{2}\\ x_{2}-x_{3}y_{2}-y_{3}z_{2}-z_{3}\\ x_{3}-x_{4}y_{3}-y_{4}z_{3}-z_{4} \end{array}\right],\\ X=\left[\begin{array}{c} x\\ y\\ z \end{array}\right],\\ B=\frac{1}{2}\left[\begin{array}{c} d_{1}^{2}-d_{2}^{2}-x_{1}^{2}+x_{2}^{2}-y_{1}^{2}+y_{2}^{2}-z_{1}^{2}+z_{2}^{2}\\ d_{2}^{2}-d_{3}^{2}-x_{2}^{2}+x_{3}^{2}-y_{2}^{2}+y_{3}^{2}-z_{2}^{2}+z_{3}^{2}\\ d_{3}^{2}-d_{4}^{2}-x_{3}^{2}+x_{4}^{2}-y_{3}^{2}+y_{4}^{2}-z_{3}^{2}+z_{4}^{2} \end{array}\right]. \end{array}$$

In indoor visible light positioning systems, the receiver to be positioned is usually located on the ground, whereas the LED emitters are all mounted on the ceiling, which is the height of the four LED emitters. Therefore, the third column element of the matrix in formula (21) is 0, because the matrix is an irreversible matrix and cannot be solved by directly transmitting the coordinate position of the receiver, so the coordinates of the receiver can be solved according to the generalized inverse concept of least multiplication. The objective function can be represented as *z*_1_=*z*_2_=*z*_3_=*z*_4_*AAX*=*A*^−1^*BX*:

(23) $$\begin{array}{c} X=\text{arg min}{\left\|AX-B\right\|}_{2}^{2}\\ =\text{arg min}{\left(AX-B\right)}^{T}\left(AX-B\right). \end{array}$$

For the convenience of representation, the squares of the two norms in formula (23) will be expressed in terms of representation, which can then be expressed as *f*(*X*):

(24) $$\begin{array}{c} f\left(X\right)=X^{T}A^{T}AX-X^{T}A^{T}B-B^{T}AX+B^{T}B. \end{array}$$

The derivative is manufactured in equation (24) and given as zero *f*(*X*):

(25) $$\begin{array}{c} \frac{\text{d}f\left(X\right)}{\text{d}X}=2A^{T}AX-2A^{T}B=0. \end{array}$$

Then the solution *X*

(26) $$\begin{array}{c} X={\left(A^{T}A\right)}^{-1}A^{T}B. \end{array}$$

#### 3.3.2. Performance Analysis of Positioning Algorithms

Positioning accuracy refers to the deviation between the estimated position of the measured target and the real position and is the most important indicator to measure the positioning performance. In positioning, the positioning accuracy in this article can be expressed as the positioning accuracy by selecting mean squared EiTor (MSE) or root mean squared error (RMSE):

(27) $$\begin{array}{c} \text{Error}=\sqrt{\left[{\left(x_{1}-x_{0}\right)}^{2}+{\left(y_{1}-y_{0}\right)}^{2}+{\left(z_{1}-z_{0}\right)}^{2}\right]}, \end{array}$$

where for the actual position coordinates of the receiver, for the estimated position coordinates (*x*_0_, *y*_0_, *z*_0_)(*x*_1_, *y*_1_, *z*_1_).

The positioning principle of relevant AOA methods is described in Figure 5.

Positioning errors caused by relevant noises are shown in Figure 6

#### 3.3.3. Positioning Principle of APIT Positioning Algorithm

In the traditional APIT positioning algorithm, there are K light sources for indoor visible light, namely S1, S2, S3, etc., SK, arbitrarily connecting three light sources S1, S2, S3, constitutes ΔS1 S2 S3. Let the unknown node be S, and the signal strength of S from the sources S1, S2, and S3 is RSS1, ＲSS2, ＲSS3. Move the unknown node S to any location near it, G1, and G1 to the source S1, S2, and S3. The signal strengths are RG1S1, RG1S2, RG1S3. If RG1S1, RG1S2, RG1S3 are greater than or less than RSS1, RSS2, and at the same time RSS3 indicates that the unknown node S is located outside of ΔS1 S2 S3, and the ΔS1 S2 S3 region is not selected as the decision area. If one of the signal strengths RG1S1, RG1S2, and RG1S3 is greater than the other two, it is smaller than RSS1 and RSS2, RSS3, or one smaller than the other two greater than RSS1, RSS2, and RSS3, indicating the unknown node S. In the interior of ΔS1 S2 S3, select the ΔS1 S2 S3 region as the judgment area, and repeat the above step C3K several times until all possible areas have been determined. Finally, the coincident area of the triangle containing the S of the unknown node is obtained, and the centroid of the polygon is found by using the centroid algorithm to find out the final positioning result.

## 4. Indoor Visible Light Positioning Algorithm Based on Compression Perception

### 4.1. Principles of Compression Perception

The theory of compression perception states that the sparsity or compressibility of a signal, as well as the selectivity of the transformation base and observation matrix, are two basic principles or important guarantees for recovering a signal from a sampling point far below the requirements of Nyquist's sampling theorem (24).

Now assuming that it is a one-dimensional discrete signal, and its table assumes that any signal in space can be uniquely represented by a set of standard orthogonal radicals, then the one-dimensional discrete signal can be represented by a linear group combination of these orthogonal radicals *xx* ∈ *R*^*N*×1^*R*^*N*^*ψ*=[*φ*_1_, *φ*_2_,…, *φ*_*N*_]*x*

(28) $$\begin{array}{c} x=\overset{x}{\underset{i=1}{\sum }}\varphi_{i}\alpha_{i}=\psi \alpha . \end{array}$$

Its tables, projection coefficients, projected sparse vectors, order orthogonal matrixes, and moments are all sparse vectors: *α*_*i*_=*x*, *φ*_*i*_*α*=*ψ*^*T*^*xψ*=[*φ*_1_, *φ*_2_,…, *φ*_*N*_]*NαxN* × 1.

Equation (28) is a sparse representation of the signal, and the equation table is the signal sparse cardinality. The original signal is projected onto an uncorrelated observation matrix of the shadow sparse matrix, resulting in observations. The process can be expressed as *xψxxψ*Φ*y*:

(29) $$\begin{array}{c} y=\Phi x. \end{array}$$

Its table, that is, the observation matrix, is the observation matrix, and the observation matrix obtained by observation is the original signal, that is, the table projection of the observation matrix on the original signal obtains a new signal representation. By compressing the observation matrix, the dimensionality of the new signal representation is already much smaller than the dimensionality of the original signal, and the amount of data obtained by Nyquist's sampling theorem is much smaller. It is obtained by substituting formula (28) into equation (29). *y*Φ*M* × *N*(*M* < *N*)*N* × 1*xM* × 1*x*Φ*yyNxM*

(30) $$\begin{array}{c} y=\Phi x\\ =\Phi \psi \alpha \\ =\Theta \alpha . \end{array}$$

In its table, for the perceptual matrix, equation (30) can be derived by solving a linear optimization problem to obtain a sparse vector, and the solution process can be expressed as Θ=Φ*ψα*:

(31) $$\begin{array}{c} \text{min}{\left\|\alpha \right\|}_{0}\text{ s.t }y=\Theta \alpha . \end{array}$$

If the signal is sparse, and if the matrix satisfies the constrained isometric properties (RIP) [50] inches, then the sparse signal can be recovered by solving the minimum norm problem by the observation matrix, which can be expressed as *xK*Φ*yl*_0_*x*:

(32) $$\begin{array}{c} x=\text{arg min}{\left\|\alpha \right\|}_{0}\text{ s.t}.\;\Phi x=y. \end{array}$$

Since equation (32) is the smallest solution, the norm is essentially an NP-hard [51] problem, which is usually converted to a problem where the norm is optimized as *l*_0_*l*_1_.

From the above description of the theory of compression perception, it can be obtained that there are three main steps of compression perception: (1) the sparse representation of the signal: (2) determine the observation matrix; (3) reconstruct the signal. Φ.

#### 4.1.1. Sparse Representation of the Signal

The Nyquist sampling theorem shows that sampling at a sampling rate twice the signal bandwidth accurately restores the original signal. However, when processing wideband signals in practice, it is often difficult to achieve due to the huge amount of computation. The theory of contraction sense shows that if a signal is sparse in a given transformation domain, it can be sampled at a rate much lower than the Nyquist sampling rate and the original signal can be accurately recovered.

The sparseness or compressibility of the signal is an important prerequisite of the theory of compression perception, fixed to a discrete-time signal of length *N*. The time-domain representation of discrete-time signal *x* is *xxx*_*n*_*n*=1,2, ⋯，*N*. Fixed to a set of canonical orthogonal bases set to the domain, as shown in equation (33), a discrete-time signal can be linearly represented by this set of canonical orthogonal roots [*φ*_1_, *φ*_2_,…, *φ*_*N*_]Ψ*x*.

(33) $$\begin{array}{c} x=\Psi s, \end{array}$$

where the matrix Ψ is *N* × *N* and *s* and *x* are both column *N* × 1 vectors. If *x* can be linearly represented by a *K*(*K* ≪ *N*) basis vector, then the signal *x* is *K* sparse. Ψ*N* × *NxsN* × 1*xK*(*K* ≪ *N*)*xK*

After a linear observation of the original dimensional signal, a dimension column vector consisting of a measured value can be obtained. The entire linear observation process is shown below *M* × *N*Φ*NxMy*_*j*_,  *j*=1,2,…, *MM*:

(34) $$\begin{array}{c} y=\Phi x. \end{array}$$

Substitute formula (33) into equation (34) to get it

(35) $$\begin{array}{c} y=\Phi x\\ =\Phi \Psi s\\ =\Theta s, \end{array}$$

where Θ=ΦΨ*M* × *N* is the perception matrix. Θ=ΦΨ*M* × *N*

#### 4.1.2. Observation Matrix

In positioning based on compression perception, a common approach is to select a sparse random matrix as the measurement matrix, which is established by each row that has only one nonzero element 1, and its column number is randomly selected from 1 to *N*. This design approach is equivalent to deploying sensor nodes completely randomly in the positioning area. This is a simple and straightforward process that can be expressed by the power measurement matrix as the product of the observation matrix, the sparse matrix, and the sparse vector in the theory of compression perception.

After sampling, compression, and encoding, the dimension of the original signal is compressed into a dimensional observation vector, that is, the dimension of the original signal is compressed as *NM*(*M* ≪ *N*)*N* − *M*.

When the observation matrix satisfies the constrained isometric condition (RIP), a definite solution exists for a system of uncertain equations. The RIP criterion is defined as follows: assume that the length of the signal is *xNK*，*ε* > 0，Θ, and that sparsity is always present in order to satisfy the perceptual matrix: *xNK*，*ε* > 0，Θ

(36) $$\begin{array}{c} 1-\varepsilon \leq \frac{{\left\|\Theta \alpha \right\|}_{2}}{{\left\|\alpha \right\|}_{2}}\leq 1+\varepsilon . \end{array}$$

Therefore, the key to the problem is how to determine whether the random projection matrix satisfies the RIP criterion. In order to reduce the complexity of this problem, the concept of correlation [even] is proposed to replace it, and the definition of relevance is as follows:

(37) $$\begin{array}{c} \mu \left(\Phi ,\psi \right)=\sqrt{n}\cdot \underset{k\geq 1,j\leq n}{\text{max}}\left|\varphi_{k},\phi_{j}\right|, \end{array}$$

where the value range *μ* is satisfied: *μ*

(38) $$\begin{array}{c} \mu \left(\Phi ,\psi \right)\in L1,\;\sqrt{n}. \end{array}$$

If there are correlated elements between the two matrices, the two matrices have a greater correlation; otherwise, they are considered less correlated.

Figure 7 shows the correlation between SIG noise ratio and LED emission power under Gaussian noise shadow.

#### 4.1.3. Signal Reconstruction Algorithms

Signal reconstruction is a very important part of compression perception theory, and without a superior reconstruction algorithm to recover the original signal, then compression perception theory has no practical effect. Signal reconstruction is the process of reconstructing the original signal from a dimensional observation vector obtained from compression, where *MyNxM* are a few common compression-aware refactoring algorithms *MyNxM*[25]:

*(1) Minimal Standard Model*. *l*_0_ From a mathematical point of view, the problem of signal reconstruction in the theory of compression perception is the problem of solving a system of uncertain equations. It can be solved by norm, as shown in equation (39) *l*_0_.

(39) $$\begin{array}{c} \text{min }{\mathrm{||}x\mathrm{||}}_{0}\text{ s.t}.\;y=\Phi x, \end{array}$$

Due to the noise present in the actual measurement, equation (40) can be converted to

(40) $$\begin{array}{c} \text{min }{\mathrm{||}x\mathrm{||}}_{0}\text{ s.t. }-\Phi {\mathrm{||}x\mathrm{||}}_{2}\leq \varepsilon . \end{array}$$

Among them, is a very small constant. Usually, the calculation of the algorithm is very unstable, and it is difficult to reconstruct the signal directly *ε*.

*(2) Minimal Standard Model*. *l*_1_ When the observation matrix [1] satisfies the RIP criterion, the norm and the norm optimization solution problem produce the same solution, so the norm solving problem can be converted to *l*_0_*l*_1_*l*_0_:

(41) $$\begin{array}{c} \text{min }{\mathrm{||}x\mathrm{||}}_{1}\text{ s.t. }y=\Phi x. \end{array}$$

Replace equation (41) with equation (4) [2], which is base distance tracking (BP) = Equation (41) is converted to

(42) $$\begin{array}{c} \text{min }{\mathrm{||}x\mathrm{||}}_{1}\text{ s.t. }y=\Phi {\mathrm{||}x\mathrm{||}}_{2}\leq \delta . \end{array}$$

In practice, the BP algorithm runs for a relatively long time.

### 4.2. Indoor Visible Light Compression Sensing Positioning

The main process of the compression perception algorithm can be described as known observation matrix and unknown signal and measurement matrix obtained through observation matrix observation, and linear observation process can be eexpressed as Φ ∈ *R*^*M*×*N*^(*M* ≪ *N*)*x* ∈ *R*^*N*^，*Y* ∈ *R*^*M*^

(43) $$\begin{array}{c} y=\Phi x. \end{array}$$

If the signal is sparse and the measurement matrix and the observation matrix meet certain conditions, the measurement matrix can be solved by a reconstruction algorithm *xKy*Φ*yx*.

Below we construct the indoor visible light positioning implementation problem as a compression perception sparse signal reconstruction problem, and the receiver is located in the positioning room, the positioning space is divided into grids, and the receiver obtains RSS measurements from the LEDs on the ceiling *NM*(*M* ≪ *N*).

Defines the receiver position information vector, as shown in equation (44). When the receiver is inside the first mesh, otherwise. Since indoor visible light positioning is only for a single target, the sparseness of the position information vector is 1. *sks*_*k*_=1*s*_*k*_=0*s*:

(44) $$\begin{array}{c} s={\left\{s_{k},\;k=1,2,\ldots ,N\right\}}^{T}. \end{array}$$

Defines a sparse matrix, as shown in equation (45), where the receiver representing the bit meter grid receives the signal power of the bit meter grid, which is located directly above the LED emitter Ψ*ψ*_*ij*_*j*(1 ≤ *j* ≤ *N*)*i*(1 ≤ *i* ≤ *N*).

(45) $$\begin{array}{c} \Psi ={\left(\begin{array}{cccc} \psi_{11} & \psi_{12} & \cdots & \psi_{1N}\\ \psi_{21} & \psi_{22} & \cdots & \psi_{2N}\\ \vdots & \vdots & \cdots & \vdots \\ \psi_{N1} & \psi_{N2} & \cdots & \psi_{NN} \end{array}\right)}_{N\times N}. \end{array}$$

Define the observation matrix, as shown in equation (46), where the first LED emitter is mounted on the ceiling above the grid, when the first LED emitter is located in the upper straight of the first grid, otherwise set. By definition, the meta-meters of a matrix of only one observation per row are set to 1, and the rest of the elements are set to 0 Φ*MNij*Φ_*ij*_=1Φ_*ij*_=0Φ.

(46) $$\begin{array}{c} \Phi ={\left(\begin{array}{cccccc} 0 & \cdots & 1 & 0 & \cdots & .\\ 0 & \cdots & 0 & 1 & 0 & \cdots \\ \vdots & . & \vdots & \vdots & . & \vdots \\ 0 & \cdots & \cdots & 0 & 1 & 0 \end{array}\right)}_{M\times N}. \end{array}$$

The matrix of measured values is shown in equation (47), where the receiver receives the optical signal emitted by the first LED and converts the optical signal into an electrical signal, which rotates from the strength of the first signal received by the LED transmitter *yM*(*M* ≪ *N*)*y*_*n*_*n*(1 ≤ *n* ≤ *M*).

(47) $$\begin{array}{c} y={\left\{y_{1},y_{2},\ldots ,y_{1N}\right\}}^{T}. \end{array}$$

According to the theory of compression perception, a matrix of measurable values is satisfied by *y*

(48) $$\begin{array}{c} y=\Phi x\\ =\Phi \Psi s\\ =\Theta s. \end{array}$$

It is transformed into a perceptual matrix Θ.

Considering the presence of measurement noise, equation (48) can be converted to

(49) $$\begin{array}{c} y=\Phi \Psi_{s}+\varepsilon \\ =\Theta s+\varepsilon . \end{array}$$

The RIP criterion is a sufficient nonessential condition for the signal to be accurately reconstructed, with a sparse position information vector of 1 degree and a quadratic measurement of that degree, which proves that when equation (50) condition is satisfied, the initial signal can be reconstructed by equation (49) with a high probability of precision *ssMMs*.

(50) $$\begin{array}{c} M\geq C\times K\times \text{log}\left(\frac{N}{K}\right), \end{array}$$

where is a small constant *C*.

Because the sparse matrix is related to the spatial domain of the observation matrix, the RIP criterion is not satisfied. In order to achieve the same effect as the RIP criterion, the selective measurement matrix is orthogonally treated ΨΦΘ=ΦΨΘ=ΦΨ*y*.

(51) $$\begin{array}{c} Y=A\Theta y\\ =A\Theta \Theta s\\ =As, \end{array}$$

where *A* is the orthogonal basis of the matrix Θ, that is, the generalized inverse of the matrix.In the case of existing noise, equation (51) can be converted to *A*Θ*A*=*orth*(Θ^*T*^)^*T*^,  Θ^+^Θ.

(52) $$\begin{array}{c} Y=A\Theta^{+}y\\ =A\Theta^{-}\Theta s+A\Theta^{-}\varepsilon \\ =As+\varepsilon , \end{array}$$

where *A* is the orthogonal matrix*A*.

This article uses the following sparse signal reconstruction algorithm to reconstruct sparse signals.

(1) The orthogonal match tracking algorithm
For the reconstruction of sparse signals, the steps of the Quadrature Match Tracking Algorithm (OMP) can be described as *Ks*
Input variables: order matrix, measured value matrix, sparseness *M* × *NAYK*
Output variable: An estimate of the sparse signal $s\hat{s}$
Initialization operation: The order matrix is represented as vector groups, support sets, and number of iterations *M* × *NA*(*a*_1_, *a*_2_,…, *a*_*N*_)*r*_0_=*Y*Λ_0_=∅*k*=1*A*_0_=[].
  Step 1: First, take the column vectors and residuals in the matrix as an inner product operation to find the column vector corresponding to the maximum absolute value of the inner product and its index value: *Aa*_*j*_*r*_*k*−1_*λ*_*k*_=arg max_*i*=1,2,⋯*N*_|*r*_*k*−1_^*T*^*α*_*j*_|
  Step 2: Update Operation: This is a collection of all the index values obtained after many iterations, which means that the sequential matrix composed of the corresponding column vectors is selected from the matrix according to the set of index values.
    (53) $$\begin{array}{c} \Lambda_{k}=\Lambda_{k-1}\cup \left\{\lambda_{k}\right\},\\ A_{k}=\left[A_{k-1},A\left(:,\lambda_{k}\right)\right],\;\Lambda_{k}kA_{k}\Lambda_{k}AM\times k. \end{array}$$
  Step 3: Solve the least squares solution:
    (54) $$\begin{array}{c} Y=A_{k}S_{k}s_{k}\\ =\text{arg min}Y-A_{k}s_{k}\\ ={\left(A_{k}^{T}A_{k}\right)}^{-1}A_{k}^{T}Y. \end{array}$$
  Step 4: Update the residuals, which represent the *r*_*k*_=*Y* − *A*_*k*_*s*_*k*_*r*_*k*_ residuals *k* obtained after iteration.
  Step 5: That is, the *k*=*k*+1 number of iterations plus 1, if yes *k* ≤ *K*, go back to step 1 to continue the iterative process, if yes *k* > *K*, stop the iteration process and perform step 6.
  Step 6: Finally, according to the correspondence with the sparse vector, an estimated recovery vector is obtained as *s*_*k*_Λ_*k*_*ss*.
(2) The greedy match tracking algorithm
The Greedy Match Tracking Algorithm (GMP) step can be described as follows:
Input variables: order matrix, measurement matrix. *M* × *NAY*
Output variable: an estimate of the sparse signal. *ss*
Initialization operation: index value collection Λ={1,2,…, *N*},  *Y*′=*Y*.
  Step 1: Find satisfaction (4.26) and is_*i*_
    (55) $$\begin{array}{c} \underset{i\in \Lambda ,s_{i}\in \left\{0,1\right\}}{\text{argmin}}{\mathrm{||}Y}^{\prime }-A{\left[0,\ldots ,0,s_{i},0,\ldots 0\right]}_{2}^{T}. \end{array}$$
  Step 2: That is, removed from the index value collection: Λ=Λ/{*i*}*i*
  Step 3: Update Residual Value: that is, the next search is done using residuals: *Y*′=*Y*′ − *A*[0,…,*s*_*i*_, 0,…0]^*T*^
  Step 4: Update the vector: *s* : *s*_*i*_=*s*_*i*_
  Step 5: Determine if the search termination condition has been reached, that is, the search is terminated, otherwise, return to step 1 to continue the search process: *s*_*i*_=0
  Step 6: Finally return the estimate of the sparse vector *ss* array
    (56) $$\begin{array}{c} y={\left\{y_{1},y_{2},\ldots ,y_{M}\right\}}^{T}. \end{array}$$

Set a reasonable threshold for the receiver's received signal strength when the direct signal of the first LED transmitter is blocked. Since the first LED emitter is located on the ceiling, directly above the first grid, set the observation matrix at this time, and set the settings as*λ*, *λy*_*i*_ < *λiij*ΦΦ_*ij*_=0*y*_*i*_=0.

### 4.3. Positioning Model

In a wireless sensor network, consider the positioning problem: *k* positions. Unknown targets are randomly distributed within a particular area; the positioning area is divided into *N* grids and assumes that the target can only be located in the center of the grid. Grid coordinates are known, so that positioning can be achieved by determining which grid the target is located in. An *N*-dimensional sparse vector *θ* represents the target location information, which contains only *k* (*k* Much less than *N*) nonzero elements, each of which corresponds to a target node, and whose corresponding ordinal number represents the grid number in which it is located. To determine the location of the target, deploy *M* sensor nodes with known locations to measure the received signal strength. Traditional positioning methods require the deployment of a sensor per mesh, which will require the deployment of a large number of sensor nodes and generate a considerable amount of work, and thus difficult to achieve. By introducing the theory of compression perception, the position vector *θ* can be accurately recovered by deploying only a small number of sensor nodes.

### 4.4. Compression Panther—Depreciation Phase

The rough positioning phase uses the compression-aware positioning algorithm proposed in section 4. The receiver is located in the positioning space, dividing the room into a discrete grid, and the receiver obtains the RSS value from the LED emitter on the ceiling. In this article, the indoor visible light positioning model has the number of meshes, the number of LED emitters, the number of meshes is 400, and the sparseness is 1, and the sample is compressed by equation (*NM*(*M* ≪ *N*)*NMNK* (57)).

(57) $$\begin{array}{c} \left[\begin{array}{c} y_{1}\\ y_{2}\\ \vdots \\ y_{M} \end{array}\right]=\left[\begin{array}{cccc} P_{1,1} & P_{1,2} & \ldots & P_{1,N}\\ P_{2,1} & P_{2,2} & \ldots & P_{2,N}\\ \vdots & \vdots & . & \vdots \\ P_{M,1} & P_{M,2} & \ldots & P_{M,N} \end{array}\right]\left[\begin{array}{c} x_{1}\\ x_{2}\\ \vdots \\ x_{N} \end{array}\right]. \end{array}$$

The *x*_*n*_=1 indicate that the target is within the grid. Determines whether the target is within the recovery range of the fence grid, and when the target is in the grid close to the fence, the positioning result is directly output. Otherwise, further fine positioning is carried out to improve the positioning accuracy, as shown in Figure 8.

Further fine localization is carried out when it is determined that the target is not within the recovery range of the grid near the perimeter wall. The precision positioning stage optimizes the multilateral measurement algorithm through the base station (LED transmitter) selection strategy, which reduces the disadvantages of the distance between the receiver and the LED transmitter, and the positioning accuracy is greatly affected by the indoor environment. During the fine positioning phase, select the nearest LED emitter of the target as the reference point for the polygon measurement.

The four LEDs are LED1, LED2, LED3, and LED4—unknown.

The distance from the target (receiver) to the LED transmitter can be calculated by the received signal strength. The calculation method of the multifaceted measurement algorithm can be expressed as follows:

(58) $$\begin{array}{c} \left\{\begin{array}{c} {\left(x-x_{1}\right)}^{2}+{\left(y-y_{1}\right)}^{2}+{\left(z-z_{1}\right)}^{2}=d_{1}^{2},\\ {\left(x-x_{2}\right)}^{2}+{\left(y-y_{2}\right)}^{2}+{\left(z-z_{2}\right)}^{2}=d_{2}^{2},\\ {\left(x-x_{3}\right)}^{2}+{\left(y-y_{3}\right)}^{2}+{\left(z-z_{3}\right)}^{2}=d_{3}^{2},\\ {\left(x-x_{4}\right)}^{2}+{\left(y-y_{4}\right)}^{2}+{\left(z-z_{4}\right)}^{2}=d_{4}^{2}. \end{array}\right) \end{array}$$

Its position represents the coordinates of the receiver position to be estimated, indicates the position of the first LED emitter, and indicates the distance from the receiver to the first LED emitter. (*x*, *y*)(*x*_*i*_, *y*_*i*_)*id*_*t*_*i*.

Equation (58) is a system of nonlinear equations that can be linearly converted to

(59) $$\begin{array}{c} AX=B, \end{array}$$

thereinto

(60) $$\begin{array}{c} A=\left[\begin{array}{ccc} x_{1}-x_{2} & y_{1}-y_{2} & z_{1}-z_{2}\\ x_{2}-x_{3} & y_{2}-y_{3} & z_{2}-z_{3}\\ x_{3}-x_{4} & y_{3}-y_{4} & z_{3}-z_{4} \end{array}\right],\\ X=\left[\begin{array}{c} x\\ y\\ z \end{array}\right],\\ B=\frac{1}{2}\left[\begin{array}{c} d_{1}^{2}-d_{2}^{2}-x_{1}^{2}+x_{2}^{2}-y_{1}^{2}+y_{2}^{2}-z_{1}^{2}+z_{2}^{2}\\ d_{2}^{2}-d_{3}^{2}-x_{2}^{2}+x_{3}^{2}-y_{2}^{2}+y_{3}^{2}-z_{2}^{2}+z_{3}^{2}\\ d_{3}^{2}-d_{4}^{2}-x_{3}^{2}+x_{4}^{2}-y_{3}^{2}+y_{4}^{2}-z_{3}^{2}+z_{4}^{2} \end{array}\right]. \end{array}$$

Since the LED emitter is considered to be on the same level as the ceiling in the actual fixed position, the third column of the matrix is usually 0. Since the matrix is irreversible, it is not possible to find the target position directly according to the least squares method, and the objective function that uses the concept of generalized inverse to solve it can be expressed as *z*_1_=*z*_2_=*z*_3_*AAX*=*A*^−1^*B*.

(61) $$\begin{array}{c} X=\text{arg min}{\left\|AX-B\right\|}_{2}^{2}. \end{array}$$

The square expansion of the two norms in equation (61) obtains it:

(62) $$\begin{array}{c} X=\text{arg min}{\left\|AX-B\right\|}_{2}^{2}=\text{arg min}{\left(AX-B\right)}^{T}\left(AX-B\right). \end{array}$$

If the squares of two norms in equation (62) are expressed as *f*(*X*), then

(63) $$\begin{array}{c} f\left(X\right)=X^{T}A^{T}AX-X^{T}A^{T}B-B^{T}AX+B^{T}B. \end{array}$$

Derivation (63) is obtained by deriving and assigning it zero *f*(*X*), then

(64) $$\begin{array}{c} \frac{f\left(X\right)}{\partial X}=2A^{T}AX-2A^{T}B=0. \end{array}$$

It can be obtained by formula (64).

(65) $$\begin{array}{c} A^{T}AX=A^{T}B. \end{array}$$

Then the solution *X*is

(66) $$\begin{array}{c} X={\left(A^{T}A\right)}^{-1}A^{T}B. \end{array}$$

Figure 9 shows the correlation between SIG noise ratio and LED emission power under Gaussian noise shadow.

### 4.5. Advantages of the Algorithm

In this article, a multitarget positioning method based on compression perception in wireless sensor networks is studied. By constructing a matrix using the received signal strength values, the position information of the signal can be represented as a sparse vector with a linear–constraint relationship with the sensor measurements. The compression sensing positioning algorithm of the visible light chamber of the mixed APIT has dramatically improved the positioning accuracy and stability.

## 5. Conclusion

Light-emitting diodes (LEDs) are one of the most promising new sources of green lighting in the twenty-first century. LED lamps and lanterns due to high efficiency, energy-saving, low price, long life, green environmental protection, pollution-free, and other advantages are widely used in lighting, display, and other fields, and LED can be used for lighting and communication characteristics, making VLC technology to become a research hotspot in recent years. In addition, with the continuous development of society, people's demand for indoor positioning services is also increasing. VLC-based indoor positioning technology has many advantages over traditional indoor positioning technology, so it has gradually become a hot topic of research.

Finally, a fusion positioning algorithm based on compression perception and multilateral measurement is proposed, which first targets the nonvisual distance of the optical signal obscured by opaque objects in the actual positioning, and the positioning error is very large, through the positioning before positioning. The preprocessor is used to reduce the impact of occlusion on the positioning. Then, in the rough positioning phase, a compression-aware positioning algorithm is used to determine the location of the mesh where the receiver is located. When the recovery position is close to the recovery range of the surrounding wall grid, there is no need for fine positioning, the positioning result is directly output, and when the receiver is not within the recovery range of the surrounding wall grid, the receiver position is accurately estimated by fine positioning. Fine positioning can reduce the impact of reconstruction errors on positioning accuracy and reduce positioning errors when the target is located near the grid boundary. The multifaceted measurement algorithm is optimized by the LED selection strategy, which can effectively reduce the positioning error of the target near the center of the room, and overcome the limitation that the positioning effect of the compression sensing positioning algorithm is not ideal when the number of LEDs is small.

## Figures and Tables

**Figure 1:** VLC indoor positioning model.

**Figure 2:** The shadow area of the triangle where the projection point *M* is located.

**Figure 3:** Projection point M is located inside the A1A2A3 Δ.

**Figure 4:** Close to the fence in two grids.

**Figure 5:** AOA method positioning principle.

**Figure 6:** Noise-induced positioning error.

**Figure 7:** Correlation between SIG noise ratio and LED transmit power under Gaussian noise shadows.

**Figure 8:** Positioning the system model.

**Figure 9:** Correlation between SIG noise ratio and LED emission power under Gaussian noise shadow.

**Table 1:** Comparison table of indoor positioning technologies.

Indoor positioning technology	Positioning accuracy	Relative cost	Merit	Shortcoming	Example
Wireless network	2–50 m	Low	Low cost and strong communication skills	Susceptible to environmental disturbances	The application adopts the placement of wireless base stations in the area, and comprehensively determines the coordinates of the Wi-Fi device to be located according to the signal characteristics of the Wi-Fi device to be located, combined with the topology of the wireless base station.
Bluetooth	2–10 m	Low	The device is small in size, easy to integrate, easy to integrate, and easy to use	The propagation distance is short and the stability is poor.	High price and less use.
Ultra-wideband	6–10 cm	Ix	High precision and strong penetration	Costly	It is mainly used in coal mines, chemicals, electric power and energy, hospitals, nursing homes, tunnels, manufacturing, public inspection and justice, and other industries.
Ultrasonic	1–10 cm	High	High positioning accuracy	The propagation distance is short and the stability is poor.	—
Radio frequency identification	0.05–5 m	Middle	The cost is not high, the precision is high	Identities have no communication skills and the distance is short.	Typical applications for personnel positioning come from the expansion of personnel attendance systems.
Siegbi	Length—2 m	Low	Low power consumption, low cost	Poor stability and susceptibility to environmental interference.	—
Infrared	5–10 m	High	High positioning accuracy	Straight line of sight, short transmission distance, easy to interfere.	It is not widely used for the time being.

**Table 2:** Positioning system parameters.

Parameter		Numeric value
Indoor environment	Reflection coefficient of the wall/ceiling/floor	0.66/0.35/0.66
	Room size	5.0 m × 5.0 m × 3.0 m
	Diffuse scale	0.7
	Specular scale	0.3

Transmitter	Coefficient of refraction	1
	LED transmit power	1 W
	Half-power angle	60°

Receiver side	Effective area	1 point × 1 point
	Sensitivity	0.4 amps/watt
	Receive the viewing angle	70°

## Data Availability

The authors do not have permission to share data from the data provider.
